# Level of consistency between students’ self-reported and observed study approaches in flipped classroom courses: How does it influence students’ academic learning outcomes?

**DOI:** 10.1371/journal.pone.0286549

**Published:** 2023-06-13

**Authors:** Feifei Han

**Affiliations:** 1 Institute for Learning Sciences and Teacher Education, Australia Catholic University, Brisbane, Australia; 2 Faculty of Education, Department of Pedagogy and Psychology, University of Hradec Králové, Hradec Králové, Czech Republic; The Hong Kong Polytechnic University, HONG KONG

## Abstract

Using Student Approaches to Learning research as a theoretical framework, the present study used both self-reported and observational log data to understand students’ study approaches in a flipped classroom course amongst 143 computer science undergraduate students. Specifically, it aimed to examine: 1) to what extent students’ study approaches identified by self-reported and observational log data are consistent with each other; and 2) to what extent students’ academic learning outcomes differ between students who showed consistent and inconsistent study approaches by self-reported and observational log data. Using The Revised Study Process Questionnaire, students were clustered as reporting either a Deep or a Surface Study Approach. Using frequencies of students’ participation in five online learning activities, they were classified as adopting either an Active or a Passive Study Approach. A 2 x 2 cross-tabulation showed a positive and moderate association between clusters of students’ study approaches resulted from two types of data. Amongst students who self-reported a Deep Study Approach, the proportion of students who adopted an Active Study Approach (80.7%) was significantly higher than those who adopted a Passive Study Approach (19.3%). In contrast, of the students who self-reported a Surface Study Approach, the proportion of students who used a Passive Study Approach (51.2%) was significantly higher than those who used an Active Study Approach (48.8%). Furthermore, students who had good study approaches by both self-report and observation did not differ from students who adopted an Active study approach by observation but reported a Surface Study Approach on course grades. Likewise, there was no significant difference in terms of academic learning outcomes between those who had poor study approaches by both self-report and observation and those who adopted Passive study approach by observation but reported a Deep Study Approach. Future studies may consider incorporating some qualitative methods in order to find out possible reasons behind the inconsistencies between self-reported and observed study approaches.

## Introduction

Over the last few decades, learning in higher education has undergone significant transformation, such as re-designing large lecture-focused courses by adopting flipped classroom courses [1]. As a special type of blended learning designs, flipped classroom courses require students to engage in “interactive content focusing on key concepts prior to class thus allowing class time for collaborative activities that clarify concepts and contextualise knowledge through application, analysis, and planning and producing solutions” [2, p. 1].

Flipped classroom courses have been widely adopted in contemporary learning design in higher education [3], as this type of course design not only promotes active learning [4], but also able to bring various benefits. To start with, flipped classroom courses are well known for their flexibility, as the online learning materials are available at any time and place so that they can easily accommodate the diverse learning preferences of students [5]. Second, flipped classroom courses are beneficial in terms of developing a number of students’ essential graduate attributes, such as problem-solving [6], interpersonal skills [7], and collaboration and teamwork skills [8]. Moreover, compared with traditional learning design, flipped classroom courses can increase students’ attendance [9], retention rates [10], as well as their learning engagement [11]. The majority of existing research has also reported better academic learning outcomes in flipped classroom courses compared with the traditional approach [12].

Compared with traditional course designs, students’ learning experiences in flipped classroom courses are highly complex as students often move back and forth between in-class and on-line learning spaces. In these experiences, students not only interact with the teaching staff and fellow students (the human elements), but also spend a significant proportion of time navigating online learning platforms where they interact with a variety of technology-enabled learning tools, such as blogs, wikis, online discussion forums, podcasts, and video clips (non-human or material elements) [13]. The complexity of learning in flipped classroom courses requires new ways and methods to be integrated into research in order to properly understand how students go about learning (study approaches).

Traditionally, research into students’ study approaches in higher education has largely relied on employing self-reported methods (e.g., self-reported questionnaires, focus groups, interviews, and dairies) [14]. However, self-reported methods and data are often criticized for their subjectivity and inability to represent the complexity of students’ contemporary learning experiences [15,16]. Moreover, self-reports are easily affected by careless answering and item nonresponse by students [17,18].

The widespread adoption of online learning management systems (LMS) and the development in the areas of learning analytics have enabled collection and analysis of observational log data in technology-mediated learning. The observational log data may not only provide relatively objective descriptions of students’ online learning, but also has potential to reflect the dynamic and nuanced differences of how students approach online learning [19].

However, fully relying on the observational log data to examine students’ study approaches without guidance from educational theories has also received criticism of being data-centric, which could result in erroneous interpretations due to a lack of sound theories and meaningful contexts [20]. To address the drawbacks of the self-reported and observational log data, in recent years, researchers have begun to employ both self-reported and observational log data to understand students’ study approach [21–24]. The present investigation will adopt Student Approaches to Learning research as a theoretical framework and will use both self-reported and observational log data to examine students’ study approaches in flipped classroom courses. The present study will expand on previous research by addressing two research gaps: 1) levels of consistency between students’ study approaches measured by self-reported and observational log data; and 2) how levels of consistency impact students’ academic learning outcomes. The following sections will review relevant literature.

### Student approaches to learning framework and self-reported study approaches

Student Approaches to Learning (SAL) research is one of the guiding frameworks widely used in higher education to understand students’ experiences of learning [25]. SAL research identifies variations in key factors of students’ experiences of learning and studies the relations between them [26]. Within SAL research framework, Biggs uses a 3P model to describe the relations of these factors by categorizing them into Presage, Process, and Product [27]. The Presage has the factors which exist prior to the time of learning in students’ learning and consists of both students’ factors (e.g., prior knowledge, personal attributes, and personality) and situational factors (e.g., institutional climate, course structure, and teaching methods). The Product concerns with various measures of students’ academic performance, such as course grades and students’ post-learning conceptions of the subject matter [28].

As to the Process, one of the main factors is how students go about learning, known as study approaches [29]. Researchers have identified qualitatively different study approaches in different academic disciplines (e.g., history, science, mathematics, biology, arts, and political sciences) and in different learning tasks (e.g., reading, writing, and learning through discussions, problem-based learning, and collaborative learning). Although specific categories of study approaches differed by disciplines and learning tasks, two broad categories of study approaches have been consistently observed [30–32], namely Surface and Deep Study Approaches. A Surface Study Approach deals with learning with minimum efforts with an intent to achieve some practical goals, such as to fulfil the compulsory requirements of the course or to pass the examination. Students taking a Surface Study Approach often report using rote memorization, a lack of independence in learning, and relying heavily on teachers’ instructions or their peers’ efforts. In contrast, students with A Deep Study Approach reports features of taking initiatives, being proactive in, and reflective of, their learning processes with a meaningful intent of learning to gain understandings [33–36].

Central to the 3P model is the relational stance [26,37], in which study approaches are not considered as stable psychological traits of learners but are simultaneously shaped by the learner and the learner’ experienced learning context [28]. Hence, learners can consciously choose different study approaches on the basis of their perceived contexts and situations of learning. The same learner may vary their study approaches in different subject matters or in different learning designs (face-to-face, online, or blended designs).

Numerous studies have been conducted to examine the relations between students’ study approaches and their academic learning outcomes since a seminal study by Säljö [38], which found students’ learning outcomes varied by the study approaches they adopted. Since then, a large number of studies have consistently identified logical relations between study approaches and academic learning outcomes that A Deep Study Approach tends to be associated with better academic learning outcomes; A Surface Study Approach tends to be related to poorer academic learning outcomes [39–42].

However, the majority of existing SAL research has used self-reports to measure study approaches, which has suffered from a number of drawbacks as mentioned above. To improve the insights of contemporary university students’ learning, suggestions have been put forward to expand the current self-reporting methods by including other types of measures to research student learning [43]. For instance, Richardson suggests that observational log data provide “both researchers and practitioners with the opportunity to monitor students’ strategic decisions in online environments in minute detail and in real time” [17, p. 359].

### Levels of consistency between self-reported and observed study approaches adopting SAL research framework

The recent development of the emerging research field of learning analytics collects rich and detailed observational log data recorded by LMS to study students’ online learning when they interact with a variety of online learning resources and activities.The observational log data has wide applications in higher education research, such as advising students’ career choice [44], detecting at risk students to improve retention [45], providing personalised feedback [46], facilitating collaborative learning [47], monitoring students’ affect in learning [48], as well as identifying learning strategies and study approaches [49,50].

There are an increasing number of studies have examined levels of consistency between using self-reported data and observational log data to understand students’ learning experiences. However, most of them have adopted either self-regulated learning [23,51,52] or learning engagement research frameworks [53]. Only two studies have specifically focused on investigating levels of consistency between self-reported and observed study approaches using SAL research framework [24,54]. However, not only did the two studies suffer from a major limitation that they relied on either self-reported data or observational log data to detect study approaches but also they produced inconsistent results.

Relying on self-reported data, Ellis et al. [54] used the Revised Study Process Questionnaire [55] to measure students’ study approaches. A hierarchical cluster analysis identified two groups of students who differed on their reporting on both Deep and Surface Scales. One cluster had significant higher ratings on the Deep Scale but significant lower ratings on the Surface Scale, hence, was referred to as reporting a Deep Study Approach. In contrast, the other cluster of students showed significant lower ratings on the Deep Scale but significant higher ratings on the Surface Scale, hence, was referred to as reporting a Surface Study Approach. The researchers then compared the observed frequencies of various types of online events between the two clusters of students and found that students reporting a Deep Study Approach participated all the online learning events significantly more frequently than those reporting a Surface Study Approach, suggesting a relatively high level of consistency between self-reported and observational log data.

However, another study by Gašević et al. only found partial consistency [24]. Gašević et al. used observational log data to detect students’ study approaches and identified four distinct study approaches, which varied on the number of sequences of the different online learning events students were engaged with. They further categorized the four study approaches into either a Deep or a Surface Study Approach according to the levels of engagement of the four study approaches. They found that students who were observed using Deep and Surface Study Approaches only differed significantly on their reporting on the Deep Scale measured by the R-SPQ [55] but not on the Surface Scale, demonstrating only partial consistency between self-reported and observational log data.

To address the limitation of the existing studies and inconsistent results, the present investigation will identify students’ study approaches using both self-reported and observational log data to see the levels of the consistency at the levels of identified groups. Furthermore, the present study will also address another research gap by examining the extent to which students’ academic learning outcomes differ between students with consistent self- and inconsistent self-reported and observational study approaches. Specifically, the following two research questions will be addressed:

1a) How do students’ observed frequencies with online learning activities and their academic learning outcomes differ by their self-reported study approaches in flipped classroom courses?
1b) How do students’ self-reported study approaches and their academic learning outcomes differ by their observed study approaches in flipped classroom courses?
1c) To what extent are students’ clusters of self-reported and observed study approaches in flipped classroom courses consistent with each other?
2. To what extent do students’ academic learning outcomes differ by levels of consistency between their self-reported and observed study approaches?

## Method

### Participants and their flipped classroom course

A cohort of 143 undergraduates who were studying towards a Bachelor of Computer Science and Information Technologies degree participated in the study. All the participants were enrolled in a flipped classroom computer science course, which lasted for 13 weeks. The face-to-face learning and teaching comprised a two-hour lecture, a two-hour tutorial, and a three-hour practice each week. Hosted in a Learning Management System (LMS), the online learning consisted of activities before and after each week’s face-to-face learning. The activities before face-to-face learning aimed to prepare for lectures, tutorials, and practice; whereas the activities after face-to-face learning aimed to consolidate and extend face-to-face learning. The following described these online activities in detail:

Online activities before face-to-face learning and teaching:

- *Pre-recorded lectures* were in video format and covered the key concepts to be discussed in the coming week’s lecture.
- *Quizzes* were embedded in video lectures and tested students’ understanding of the contents in the pre-recorded lecture.
- *Readings* were in pdf format and covered essential readings for each week.

Online activities after face-to-face learning and teaching:

- *Exercises* were in multiple-choice format and tested students’ understanding of the key concepts in each week.
- *Problem-solving questions* were in open-ended format and assessed students’ abilities to apply theories to solve practical problems.

### Instruments and data

#### The revised study process questionnaire to collect self-reported study approaches

We used the R-SPQ to collect the students’ self-report study approaches. The R-SPQ has 20 items, with 10 items being the Deep Scale and 10 items being the Surface Scale [55]. However, the Confirmatory Factor Analysis of the two-factor solution with 20-items did not show satisfactory fit of the data: χ^2^ = 342.46, *p* = .00, CFI = .82, TLI = .80, RMSEA = .08. By removing 2 cross-loading items in each factor, the final retained 16 items demonstrated appropriate fit: χ^2^ = 163.84, *p* = .00, CFI = .92, TLI = .91, RMSEA = .07. The Cronbach’s alpha reliability of the Deep and Surface Scales were .82 and .86 respectively.

#### The learning management system (LMS) to collect observed frequencies of students’ learning online activities

We used the analytic functions in the LMS to collect the observed frequencies of five types of online learning activities, namely pre-recorded lectures, quizzes, readings, exercises, and problem-solving questions.

#### Students’ academic learning outcomes

We used course grades as students’ academic learning outcomes. The maximum course grades were 100, consisting of: course preparation (maximum 20); the practice project (maximum 20), and the close-book examination (maximum 60).

### Ethical consideration and data collection

Before the data collection, ethics was applied and granted by the ethics committee of the researcher’s university. We strictly followed the ethical procedures which required written consent from all the participants, who agreed to voluntarily complete the questionnaire, to allow access to log data in LMS and course grades. The questionnaire data were collected towards the end of the semester in students’ practice sessions and the observational log data and course grades were collected upon the completion of the course.

### Data analysis

To answer the research question 1a, we conducted two separate hierarchical cluster analyses using either self-reported data or observational log data respectively. For the self-reported data, we used the mean scores of the Deep and Surface Scales to cluster students. On the basis of cluster membership, a series of one-way ANOVAs were performed to examine if there were significant differences in the frequencies of observational log data and course grades. We then conducted a second hierarchical analysis using the mean scores of frequencies of five online learning activities to cluster students. Similarly, based on cluster membership, one-way ANOVAs were conducted to investigate if students differed in their self-reported study approaches and course grades (to answer research question 1b). For research question 1c, we conducted cross-tabulation using students’ clusters resulted from the two above-mentioned hierarchical cluster analyses to examine levels of consistency between self-reported and observed study approaches.

To answer the second research question, first we categorized students into four groups: 1) poor study approaches by both self-report and observation; 2) poor observed study approaches but good self-reported study approaches; 3) good observed study approaches but poor self-reported study approaches; and 4) good study approaches by both self-report and observation. We then compared students’ academic learning outcomes between groups using a one-way ANOVA. Because of the small sample size, power analyses were also conducted for all the one-way ANOVAs.

## Results

### Results of research question 1a –differences in students’ observed frequencies of online learning activities by their self-reported study approaches

The hierarchical cluster analysis using the mean scores of the Deep and Surface Scales identified a two-cluster solution of 57 and 86 students in each cluster respectively (see Table 1). The one-way ANOVAs showed significant differences on their self-reported study approach: Deep Study Approach (*F*(1, 142) = 110.03, *p* < .01, η^2^ = .44); and Surface Study Approach (*F*(1, 142) = 22.28, *p* < .01, η^2^ = .14). Cluster 1 students reported significantly higher ratings on Deep Scale but lower ratings on the Surface Scale than cluster 2 students. Hence cluster 1 students reported a Deep Study Approach and cluster 2 students reported a Surface Study Approach respectively. In terms of the observed frequencies of online learning activities between students reported a Deep and a Surface Study Approach: the one-way ANOVAs found that out of five online learning activities, they differed significantly on three of them: readings (*F*(1, 142) = 6.59, *p* < .05, η^2^ = .05); exercises (*F*(1, 52) = 4.05, *p* < .05; η^2^ = .03); and problem-solving questions (*F*(1, 142) = 7.39, *p* < .05, η^2^ = .05). So did the final grades (*F*(1, 142) = 4.55, *p* < .05, η^2^ = .05). Students reported a Deep Study Approach were also found to participate in these three online learning activities significantly more frequently and to obtain significantly higher course grades than students reported a Surface Study Approach. The results of power analyses of all the significant results were above .70, except for frequencies of exercises (.52) and course grades (.56), which also showed small effect sizes (η^2^ = .03 and η^2^ = .05 for frequencies of exercises and course grades respectively). These results suggest that in order for large effect sizes to be detected for differences on frequencies of exercises and course grades with 70% of power and with alpha at .05 between the two clusters of students, a larger sample size is required.

**Table 1:** Observed frequencies of online learning activities by different self-reported study approaches.

variables	Deep Study Approach: 57		Surface Study Approach: 86		*F*	*p*	η^2^	observed power
	*M*	*SD*	*M*	*SD*				
*self-reported data*								
Deep Scale	5.40	0.81	4.04	0.72	110.03	**.00**	.44	1.00
Surface Scale	2.84	1.41	3.70	0.77	22.28	**.00**	.14	1.00
*observational log data*								
lectures	363.28	363.31	322.50	420.81	0.36	.55	.00	.09
quizzes	271.35	729.93	134.48	130.20	2.90	.09	.02	.39
readings	906.16	462.52	727.88	365.13	6.59	**.01**	.05	.72
exercises	291.51	414.18	188.98	185.54	4.05	**.04**	.03	.52
questions	3059.02	1574.33	2430.79	1185.06	7.39	**.01**	.05	.77
*academic learning outcomes*								
course grades	68.91	18.33	63.11	14.14	4.55	**.04**	.05	.56

### Results of research question 1b –differences in students’ self-reported study approach by their observed study approach

The hierarchical cluster analysis using observational log data also produced a two-cluster solution, which had 88 and 55 students respectively (see Table 2). The one-way ANOVAs showed significant differences on the frequencies of all five online learning activities between the two clusters: pre-recorded lectures (*F*(1, 142) = 36.78, *p* < .01, η^2^ = .21); quizzes (*F*(1, 142) = 6.29, *p* < .01, η^2^ = .04); readings (*F*(1, 142) = 97.83, *p* < .01, η^2^ = .41); exercises (*F*(1, 142) = 22.78, *p* < .01, η^2^ = .14); and problem-solving questions (*F*(1, 142) = 117.17, *p* < .01, η^2^ = .45). Cluster 1 students were observed to participate in all the five online learning activities significantly more frequently than cluster 2 students. Therefore, cluster 1 and cluster 2 students adopted an active study approach and a passive study approach respectively.

**Table 2:** Self-reported study approaches by clusters of different observed study approaches.

variables	Active Study Approach: 88		Passive Study Approach: 55		*F*	*p*	η^2^	observed power
	*M*	*SD*	*M*	*SD*				
*observational log data*								
lectures	481.39	445.80	110.55	101.47	36.78	**.00**	.21	1.00
quizzes	266.24	590.67	65.51	61.27	6.29	**.00**	.04	.70
readings	1007.95	377.21	464.53	193.77	97.83	**.00**	.41	1.00
exercises	318.37	351.77	88.20	78.67	22.78	**.00**	.14	1.00
questions	3415.33	1250.31	1506.60	478.87	117.17	**.00**	.45	1.00
*self-reported data*								
Deep Scale	4.79	0.99	4.25	0.95	10.27	**.00**	.07	.89
Surface Scale	3.25	1.20	3.54	1.06	2.17	.14	.02	.31
*academic learning outcomes*								
course grades	70.57	14.71	57.18	14.96	27.66	**.00**	.16	1.00

The results of one-way ANOVAs further showed that students who used an Active Study Approach also reported significant higher ratings on the Deep Scale (*F*(1, 142) = 10.27, *p* < .01, η^2^ = .07); and had significant higher grades (*F*(1, 142) = 10.27, *p* < .01, η^2^ = .07) than students who employed a Passive Study Approach. However, the two clusters of students did not differ on their reporting on the Surface Scale. The results of power analyses of all the significant results were above .70.

### Results of research question 1(c)–consistency between self-reported and observed study approaches

The results of the cross-tabulation demonstrated a significant and moderate association between the cluster membership results from the self-reported and observed study approaches: χ^2^(1) = 14.71, *p* < .01, φ = .32. Table 3 shows that amongst students who self-reported a Deep Study Approach, the proportion of students who adopted an Active Study Approach (80.7%) was significantly higher than those who adopted a Passive Study Approach (19.3%). In contrast, of the students who self-reported a Surface Study Approach, the proportion of students who used a Passive Study Approach (51.2%) was significantly higher than those who used an Active Study Approach (48.8%).

**Table 3:** Results of the cross-tabulation.

clusters	count % within observed approach	Active Approach	Passive Approach	total
Deep Approach	count	46_a_	11_b_	57
	% within observed approach	80.7%	19.3%	100.0%
Surface Approach	count	42_a_	44_b_	86
	% within observed approach	48.8%	51.2%	100.0%
total	count	88	55	143
	% within observed approach	61.5%	38.5%	100.0%

*Note*: Different subscript letters denote a subset of self-reported study approaches whose column proportions differ significantly from each other at the .05 level.

### Results of research question 2 –academic learning outcomes by levels of consistency between self-reported and observed study approaches

The results of one-way ANOVA revealed that students in four groups (i.e., group 1 –poor study approaches by both self-report and observation: n = 44; group 2 –poor observed study approaches but good self-reported study approaches: n = 11; group 3 –good observed study approaches but poor self-reported study approaches: n = 42); and group 4 –good study approaches by both self-report and observation: n = 44) differed significantly on their academic learning outcomes (*F*(3, 142) = 10.69, *p* < .01, η^2^ = .19). The power analysis showed an observed power of 1.00. The pairwise post-hoc comparison showed that group 4 students (who had good study approaches by both self-report and observation) and group 3 students (who had good observed study approaches but poor self-reported study approaches) obtained significantly higher grades than group 2 students (who had poor observed study approaches but good self-reported study approaches) and group 1 students (who had poor study approaches by both self-report and observation). However, there were no significant differences either between students in group 4 and group 3 or between students in group 2 and group 1.

## Discussion

The present study examined: 1) the consistency between students’ self-reported and observed study approaches in flipped classroom courses adopting a SAL research framework; and 2) students’ academic learning outcomes by the levels of consistency between their self-reported and observed study approaches.

### Consistency between self-reported and observed study approaches

We detected students’ study approaches using both self-reported and observational log data. No matter we used self-reported or observational log data to identify study approaches, the other type of data only showed partial consistency. Between the two clusters of students reporting a Deep and Surface Study Approach, they only differed on the frequencies of participation in three out of five online learning activities, namely readings, exercises, and problem-solving questions. One possible reason why the two clusters of students did not differ on frequencies of pre-recorded lectures and quizzes (which tested students’ understandings of the lectures) could be completion of quizzes contributed to 20% of the course grades.

Between the two clusters of students who adopted an Active and a Passive Approach, they only differed on the Deep Scale but not the Surface Scale. In addition, the partial consistency results were further supported by the moderate association between student clusters resulted from the self-reported and observed study approaches. Our results of partial consistency results aligned with the results in Gašević et al [24].

However, students’ academic learning outcomes showed a consistent pattern irrespective to using which types of data to identify students’ study approaches. We found students who reported a Deep Study Approach scored significantly highly than their peers who reported a Surface Study Approach. Similarly, students who were observed more active in online learning also obtained significant better grades than their counterparts who were observed less active in online activities.

### Academic learning outcomes by levels of consistency between self-reported and observed study approaches

In this study, we found that the less than two thirds (61.5%) of students’ study approaches were consistent between how they reported the learned and how they were observed to learn. In a study by Ye and Pennisi on levels of consistency between students’ self-regulated learning strategies by self-reports and observation, the results showed less than two thirds of students in the consistent groups (from 30.8% to 53.9% depending on whether there were three or two types of self-regulated learning strategies) [23].

Of the rest of students (38.5%) in the two inconsistent groups, the majority of them were in the group of good observed study approaches but poor self-reported study approaches (29.4%). Furthermore, the two consistent groups of students who had either better or poorer study approaches as reflected by both self-reported and observational log data also obtained higher and lower course grades respectively. Furthermore, our results showed that students who had good study approaches by both self-report and observation (group 4) did not differ from students who adopted a good study approach by observation but reported a Surface Study Approach (group 3) on course grades. Likewise, there was no significant difference in terms of academic learning outcomes between those who had poor study approaches by both self-report and observation (group 1) and those who adopted less desirable online study approaches by observation but reported a Deep Study Approach (group 2). The qualitative results of Ye and Pennisi’s [23] study revealed that students with poor monitoring and self-reflection abilities (identified as poor self-regulated learners) were less accurate in terms of reporting their learning. However, as the present study did not use qualitative methods, it was unknown the reasons of the inconsistencies between self-reported and observed study approaches among the participants.

### Limitations and directions for future research

Some limitations of the study need to be pointed out so that future research design can improve on these. To start with, the sample size of the study was small and the recruitment only focused on a single discipline–computer science. Previous research has shown disciplinary variations in terms of the preferred study approaches. For instance, a recent study by Ng and Yong [56] compared study approaches used by undergraduates from two science disciplines and found that biosciences undergraduates tended to report deep approaches, whilst a higher proportion of pharmacy undergraduates reported surface approaches. Ng and Yong’s study only used self-reported data to measure study approaches across disciplines. Future research may combine both self-reported and observational log data to examine study approaches of students from diverse disciplines for possible disciplinary variations to be discovered. Second, the R-SPQ is a commonly used self-reported instrument in the SAL research framework, it does not make a clear distinction between students’ study approaches in the face-to-face and online components. However, the observational log data was concerned with the online part of the learning in the flipped classroom course. Future studies should use a self-reported questionnaire which can clearly distinguish between how students go about learning in-person and online. Furthermore, the present study only used one type of observational log data–frequency to examine students’ observed study approaches. The advancement of learning analytics functions has made it possible to record a diversity of types of log data, such as time spent on different types of online learning activities (duration), the exact time at which a logged event occurs (timestamp), and the sequences of online events (sequence) [22,57–59]. Therefore, future studies may employ multiple types of log data to examine students’ observed study approaches [49,50]. An additional limitation for future research to address is to examine possible reasons behind the two inconsistent groups, namely students with good observed study approaches but poor self-reported study approaches and students with poor observed study approaches but good self-reported study approaches. Future studies can use qualitative methods, such as interviews, to find out why there is a mismatch between how students’ reported their study approaches and what they actually did in learning.

## Conclusion

The present study adopted the framework of Student Approaches to Learning research to compare levels of consistency of study approaches measured by a self-reported questionnaire and log data extracted from LMS among a cohort of Australian computer science undergraduates in a flipped classroom course. It also examined students’ academic learning outcomes of students who showed consistent and inconsistent study approaches by self-reports and observation. A positive and moderate association was found between students’ self-reported and observed study approaches. Students’ academic learning outcomes also differed by levels of consistency between their self-reported and observed study approaches. Due to the quantitative nature of the study, it was unknown the reasons of the inconsistencies between self-reported and observed study approaches, which may be revealed by combining quantitative and qualitative methods in future research.
